# Improved Interactive Genetic Algorithm for Three-Dimensional Vase Modeling Design

**DOI:** 10.1155/2022/6315674

**Published:** 2022-07-08

**Authors:** Dongbo Huang, Xing Xu, Yinglong Zhang, Xuewen Xia

**Affiliations:** ^1^School of Computer Science, Minnan Normal University, Zhangzhou 363000, China; ^2^School of Physics and Information Engineering, Minnan Normal University, Zhangzhou 363000, China

## Abstract

Interactive genetic algorithm (IGA) is an effective way to help users with product design optimization. However, in this process, users need to evaluate the fitness of all individuals in each generation. It will cause users' fatigue when users cannot find satisfactory products after multi-generation evaluations. To solve this problem, an improved interactive genetic algorithm (IGA-KDTGIM) is proposed, which combines K-dimensional tree surrogate model and a graphic interaction mechanism. In this algorithm, the K-dimensional tree surrogate model is built on the basis of users' historical evaluation information to assist the user's evaluation, so as to reduce the times of users' evaluation. At the same time, users are allowed to interact with the graphic interface to adjust the shape of the individual, so as to increase users' creation fun and to make the evolution direction of the population conform to users' expectations. The IGA-KDTGIM is applied to the 3D vase design system and independently experimented with IGA, IGA-KDT, and IGA-GIM, respectively. The average fitness, maximum average fitness, and evaluation times of statistical data were compared and analyzed. Compared with traditional IGA, the number of evaluations required by users decreased by 60.0%, and the average fitness of the population increased by 15.0%. The results show that this method can reduce the users' operation fatigue and improve the ability of finding satisfactory solutions to a certain extent.

## 1. Introduction

With the rapid development of the market, customer-centered product customization has become increasingly important [1]. However, product customization poses great challenges to customers' professional knowledge and design ability. Interactive genetic algorithm (IGA) [2, 3] is a very effective method to help customers design products. It is also a good way to integrate products and people's ideas, finally obtaining the optimal solution suitable for users through genetic evolution.

IGA is developed from genetic algorithm (GA). GA is a feasible method to optimize the performance index of explicit objective. GA has been involved in the optimization of target systems, models, and performance in multiple domains. Recently, GA has been applied to fluid dynamics [4], non-linear corneal shape model [5], non-linear reactive transport model [6], non-linear electric circuit models [7], solving the singular three-point second-order boundary value problems [8], non-linear COVID-19 disease system [9], and second-order Lane–Emden equations in astrophysics [10]. These applications will inspire researchers to use GA to solve potential problems in related fields. As IGA has many similar characteristics with GA, with the development of GA, IGA will be promoted.

The IGA is an evolutionary optimization algorithm based on human-computer interaction, which realizes the intervention and guidance of the evolutionary process to solve a class of implicit performance index optimization problems that cannot be solved by traditional GA. At present, IGA has achieved great success in image retrieval [11], clothing design [12], music creation [13], and product modeling design [14]. However, the traditional IGA also has some shortcomings. The algorithm integrates the factors of thinking and emotion, knowledge background, and personal preference into the individual evaluation, which leads to the uncertainty of the individual fitness and non-unique optimization results. In the IGA, the evolution of the population has a certain degree of randomness. Since the users only need to evaluate the fitness of the individual, IGA reassembles the population features according to the fitness of the individual to produce the next generation. This evolution process does not follow the users' thinking, so the next generation produced by such a process does not always conform to the user's aesthetics. As a result, users often need to evolve for multiple generations. In the process of small population evolution, it is easy for the traditional IGA to fall into the local optimal solution, and there is no other escape mechanism to disperse the population into another solution space, so it is difficult for the population to jump out of the local optimal solution. Every population evolution needs to get the fitness evaluation of users. However, frequent user evaluation will make users feel tired easily.

To overcome the above shortcomings, an improved IGA (IGA-KDTGIM) that combines K-dimensional (K-D) tree [15] surrogate model and graphic interaction mechanism [16] has been proposed. This method builds a K-D tree model based on the historical data of users' evaluation and predicts the fitness of new individuals through the model to assist users in evaluation. If the predicted fitness does not meet the user's expectations, the user can make adjustments. Adjusting the fitness of the individual will save the data for the next update of the surrogate model. When the user has specific requirements for individual features, they can adjust individuals through the graphic interaction mechanism, helping themselves to speed up the search for satisfactory solutions. The advantage of this method is that building surrogate models can predict individual fitness and help user's evaluation, so as to reduce user fatigue. On the basis of evaluation interaction, increasing the way of graphic interaction can improve the fun of the user in the process of creation, avoid the fatigue caused by users' frequently repeated operations, and improve the user's satisfaction.

At present, IGA has achieved positive results in relieving the fatigue of users. Many researchers have used surrogate models to predict the fitness of evolutionary individuals, thereby reducing the burden of evaluation. Gong et al. [17] used the knowledge of users with similar preferences to construct a surrogate model based on the nearest neighbor collaborative filtering algorithm. Sun et al. [18] used support vector regression machine as a surrogate model to approximate user's cognition. Due to the uncertainty of the users' perception of the population, it is difficult to express the fitness of an individual with precise numbers. Therefore, some researchers use fuzzy numbers and interval ranges to express the fitness, thereby improving user evaluation efficiency and reducing users' fatigue. Gong et al. [19, 20] proposed adaptive IGA with individual interval fitness and IGA with individual fuzzy fitness. Dou et al. [21] proposed an IGA with interval individual fitness based on hesitancy.

Many researchers have introduced the distributed IGA and collaboration between users, to improve the efficiency of optimization. Miki et al. [22] proposed a global asynchronous distributed IGA. Fukumoto et al. [23] proposed a parallel distributed IGA. Guo et al. [24] introduced the multi-user collaboration strategy to predict the interval fitness of individuals by using similar individuals and sharing similar users, making full use of the advantages of group decision making. Sun et al. [25] proposed a Boolean evaluation method which used the selection method to replace the user's scoring and reduce user's operations. Hao et al. [26] proposed an extinction mechanism to reduce the search space and improve the efficiency of IGA search.

Although there are still many methods [27, 28] proposed to optimize the performance of the IGA, in traditional IGA, the uncertainty of user's cognition and the randomness of evolutionary individuals will lead to inaccurate fitness of individual evaluation, and the few satisfactory solutions generated by evolution will lead to low optimization efficiency and much user fatigue. At present, IGA interacts mainly by evaluating the fitness of individuals, and there is relatively little research on the direct interaction with individual features.

This research is carried out from the following objectives. The feasibility was verified by applying IGA-KDTGIM to the 3D vase modeling design system. The KDT is introduced to study its prediction accuracy and help users reduce the number of evaluations. The GIM was introduced to study its effect on user evaluation fitness. The innovative contribution of the algorithm and application system designed in this paper in exploring its performance is reflected in the following. First, the KDT model is based on the nearest neighbor search algorithm to predict the fitness of the population, so as to improve the user's evaluation efficiency and reduce the user's fatigue. Second, the GIM is introduced to expand the population search range and avoid premature convergence, thereby improving population fitness. Third, the proposed algorithm is applied to the 3D vase modeling design system, in which the vase model is constructed by parameterization and the parameter accuracy is improved, so that the feasibility, accuracy, and stability of the algorithm are recognized in the system.

### 1.1. The Proposed Method

This interactive algorithm is based on an IGA combined with a K-D tree surrogate model, and it predicts the fitness of an individual through similar individuals to help users recognize individuals and reduce the number of boring evaluation operations. In order to enable users to better participate in product design, the graphic interaction mechanism is added to the algorithm. Through this mechanism, users can modify their individual features, accelerate IGA's search for user satisfaction solutions, and improve their satisfaction. The method implementation is described in the following section.

### 1.2. K-Dimensional Tree Principle

The K-D tree, which can divide the existing data in consequent space, is a K-dimensional index data structure. It divides each parent node in the tree into two subspaces, and the subspace is divided until the subspace cannot be divided any more, thereby forming different subspaces. Each node in the tree corresponds to a K-dimensional hyperrectangular region which becomes the subspace of the search point when the search point is located.  Figure 1 shows the data division diagram of 20 points in K-D tree when *K* = 2. The description of K-D tree is divided into two parts: tree construction and search.

The construction of K-D tree mainly divides the multi-dimensional dataset into a binary tree. In order to make a more balanced and reasonable division of the space by each dimension, the space would be divided according to the dimension with the largest variance. When dividing in a certain dimension, the median is used as the dividing value to make the number of nodes in the left and right subtrees as consistent as possible. The structure of the K-D tree is as follows:

1. Performing variance calculation on each dimension of the dataset and selecting the dimension with the largest variance to divide the dataset.
2. Dividing the dataset into two subsets according to the median of the selected dimension. Those less than the median are classified into the left subset, and those greater than the median are classified into the right subset.
3. Repeating the above two operations for each subset until the subset cannot be divided.

The searching of nearest neighbor of K-D tree [29] is an important part of the similarity matching of two instances. The distance between two instance points in the feature space can reflect the similarity between the two instances. The normalized Euclidean distance measure can be used to calculate the distance between two instance points. The data of normalization expression are as follows:

(1) $$\begin{array}{c} x^{\prime }=\frac{x-\min\left(x\right)}{\max\left(x\right)-\min\left(x\right)}. \end{array}$$

The expression for the Euclidean distance is defined as follows:

(2) $$\begin{array}{c} d\left(x,y\right)=\sqrt{\sum_{i=1}^{n}{\left(x_{i}-y_{i}\right)}^{2}}. \end{array}$$

The method of binary search is used to search for the nearest similarity starting from the root node. If the searched point is less than the value of the current node, enter the left subtree; otherwise, enter the right subtree, until the child node is a leaf node. The searched leaf node is saved as the current nearest node, and then each node is recursively backtracked, and the subtree node on the other side is checked to see if there are any closer nodes. The distance from node to the search point is calculated and compared with the distance from the current nearest node to the search point. If there is a node that is closer than the currently saved nearest neighbor node, update that node to the current nearest neighbor node. When the search reaches the root node, the search will be terminated to get the nearest neighbor node.

### 1.3. Data Acquisition and Update

Since the surrogate model is used to approximate the user's evaluation, it usually requires a large number of evaluation samples of the users to meet the accuracy of the model. Only collecting limited data on the current user will undoubtedly increase the user's fatigue. Therefore, this research has collected a large number of online user evaluation data, including user information data, individual characteristic parameters, and fitness. A K-D tree model has been constructed from the historical evaluation data of similar users, and the fitness of similar individuals of similar users can be quickly found by this model, which can be used as the fitness of new individuals.

Since the prediction of the surrogate model is based on the evaluation information of similar users, the predicted adaptive values may be inconsistent with the evaluation of users. Therefore, users are allowed to modify and submit the individual fitness predicted by the surrogate model, and then the data evaluated by the users will be saved. Since updating the surrogate model is a time-consuming process, to avoid affecting the user design experience, the system will automatically update the surrogate model when the population evolution is being terminated by the user.

### 1.4. Graphic Interaction Mechanism

In traditional IGA, population evolution has a certain degree of randomness because population evolution does not exchange two specific features or generate new specific features according to the user's wishes. If a user wants an individual with a specific feature, but the population does not, the user will have to go through more generations of evolution before the individual with this feature appears, resulting in increased evolutionary generation and low efficiency. The randomness of population evolution is mainly manifested both in the randomness of population initialization and the uncertainty of individual mutation. In traditional IGA, each individual in the initial population is generated by a random combination of features by the computer system. Different initial population contains individuals with different features, and the features favored by users will also appear randomly. The operation of individual mutation is the operation of individual gene sequences by the mutation operator, and then it is difficult for the mutation operator to operate according to the degree of users' preference.

To solve the above problems, a graphic interaction mechanism has been proposed. This method allows users to modify individual features according to their own preferences, so that the population can quickly mutate according to users' expectations. Considering that most users are non-designers, computer graphics [30] have been integrated and parameterization has been adopted to construct 3D models.  Figure 2 shows the graphical interactive interface. The left side is a 3D model of the individual, and the right side shows the parameters that control the individual features. Through this interface, users only need to control the feature parameters, and the system will automatically change the shape of the individual. Through this way, users can modify the features of individual dissatisfaction and add them into the population. When the population falls into the local optimum, users can jump out of the local optimum and increase the diversity of generations through this mechanism.

### 1.5. Algorithm Process

This algorithm process has been improved based on the idea of IGA. The surrogate model was constructed to predict the fitness of each generation of individuals. The user can modify the dissatisfaction with fitness and ensure the individual's fitness in line with his expectations. When the population has evolved to the 10th generation or more, users are allowed to adjust the shaping of individuals according to their own preferences. Due to the user's unfamiliarity with the evolving individual in the early stage of evolution, the graphical interaction mechanism was set after the 10th generation When the user modifies the fitness of an individual, the new evaluation data will be saved at the same time, which is convenient for the next update of the surrogate model and makes its prediction results more reasonable. The algorithm process is shown in Figure 3. Algorithm 1 shows the pseudocode for the details of the algorithm steps.

### 1.6. Construction of the Vase Design System

Vases, the common decoration for furniture, have a beautiful appearance and come in a variety of shapes. This vase design system changes the shape and texture of the vase and is displayed to users in a 3D form, which makes vases more diverse and realistic. Combined with the algorithms in this paper, users can design the vase according to their personal preferences, and the design speed has been improved to a certain extent. The design of the system consists of three main parts: parameter setting, vase structure and coding, and interactive interface.

### 1.7. Parameter Setting

In order to better improve the efficiency of customer design and reduce the fatigue of users, it may be particularly important to reasonably set the population size and terminal generation. Therefore, the population size of the system is set to 6, and the termination number of evolution generations is set to 20. When the system detects that the evolutionary generation has reached the 20th generation, it will automatically terminate. As for the selection of operator, IGA applies the random sampling selection and the elite strategy, in which the crossover operator and mutation operator use two-point crossover and simple mutation method, respectively.  Figure 4 shows the operation method of crossover and mutation. When a pair of genes crosses, the segments of two gene sequences will exchange. When a gene is mutated, some of its sequences will be reversed. The crossover probability is set as 0.9, and the mutation probability is set as 0.1.

### 1.8. Vase Construction and Coding

In order to make the vase design more flexible, a modeling method based on bicubic Bezier surface [31] has been used. This method draws the grid model of the 3D cylindrical coordinate points. Then, by adjusting the control point parameters, various vase grid models are generated. Bicubic Bezier surfaces are defined as follows:

(3) $$\begin{array}{c} p\left(u,v\right)=\overset{3}{\underset{i=0}{\sum }}\overset{3}{\underset{j=0}{\sum }}P_{i,j}B_{i,3}\left(u\right)B_{j,3}\left(v\right),\left(u,v\right)\in \left[0,1\right]\times \left[0,1\right], \end{array}$$

where *B*_*i*,3_(*u*) and *B*_*j*,3_(*v*) are basis functions and *P*_*i*,*j*_ belongs to a 3 × 3 two-dimensional grid of control points. Expansion equation:

(4) $$\begin{array}{c} p\left(u,v\right)=\left[\begin{array}{cccc} u^{3} & u^{2} & u & 1 \end{array}\right]\left[\begin{array}{cccc} -1 & 3 & -3 & 1\\ 3 & -6 & 3 & 0\\ -3 & 3 & 0 & 0\\ 1 & 0 & 0 & 0 \end{array}\right]\left[\begin{array}{cccc} p_{0,0} & p_{0,1} & p_{0,2} & p_{0,3}\\ p_{1,0} & p_{1,1} & p_{1,2} & p_{1,3}\\ p_{2,0} & p_{2,1} & p_{2,2} & p_{2,3}\\ p_{3,0} & p_{3,1} & p_{3,2} & p_{3,3} \end{array}\right]\left[\begin{array}{cccc} -1 & 3 & -3 & 1\\ 3 & -6 & 3 & 0\\ -3 & 3 & 0 & 0\\ 1 & 0 & 0 & 0 \end{array}\right]\left[\begin{array}{c} v^{3}\\ v^{2}\\ v\\ 1 \end{array}\right]. \end{array}$$

The vase model consists of three parts: the mouth, the body, and the bottom. Since the vase approximates a cylinder, a bicubic Bezier surface can form a quarter surface. Therefore, the splicing of four bicubic Bezier surfaces can represent the body of revolution. The body of the vase consists of eight bicubic Bezier surfaces, and both the opening and bottom of the vase include four surfaces. It is possible to adjust the shape of the vase by adjusting the control points of the curved surface. The mesh model of the vase surface is shown in Figure 5.

In order to make the vase model more realistic and diverse, the texture image of the vase has been pasted to the surface of the vase model by using image texture mapping [32]. The parameters of the definition domain of each surface are, respectively, *u*, *v* which determine the spatial coordinates of the surface. The parameters of the image are also *u*, *v*. When the texture of a certain point on the surface needs to be read, the texture color of the point can be obtained by querying the corresponding texture elements of the image with the *u* and *v* bilinear interpolation results of the surface as coordinates. The model of the vase with texture mapping is shown in Figure 6.

The system encodes three parts of the vase: the surface, the height, and the texture map. Different gene sequences represent different vases. Because the vase is a central rotating symmetrical body, the outline of the vase body surface is represented by two cubic Bezier curves [33]. As shown in Figure 7, the curve of the vase body consists of feature points P1 to P7. The curve of the body of the vase consists of anchor points (P1, P4, P7) and control points of curvature (P2, P3, P5, P6). The height of the vase is another an important feature. The vertical structure of the model has been modified to make the vase different in height.

The gene code of the vase is also composed of the three features mentioned above, and it adopts binary code string. P1–P7 genes of the vase control points were all 8 bit, representing the continuous range from 0 to 2.55 multiplier when the abscissa of the control points was amplified. The gene of the vase height is also 8 bit, and its value range is the same as the control point of the vase body, indicating that the ordinate is magnified. The texture has 6 bits, indicating that the number of the pictures is from 0 to 63. If more texture pictures have been used, longer bits should be used to represent the texture picture coding. Therefore, the main gene of the vase is 70 bits, and different vases can be produced by changing the gene position. After the evolvement of individuals, the corresponding individual of the solution can be obtained through decoding and displayed to the user.

### 1.9. Interaction Interface

In this system, a system interaction interface has been provided for the users, as shown in Figure 8. The interface displays each generation population with a 3D model, and the displayed vases will automatically rotate, which is convenient for users to observe the texture and the shape of the vase. At the same time, the user can also operate the vase by rotating, magnifying, and moving, which helps the user to observe all parts of the vase. Each vase has its own scoring area, and the scoring value ranges from 0 to 10, indicating satisfaction (0 means not satisfied and 10 means the most satisfied).

After evolution of the 10th generation, the user can click on the vase to modify it. The user can check the parameters of the vase and adjust the parameters of the vase by using the slider. Meanwhile, the vase model will be changed dynamically as the parameters change, as shown in Figure 2.

### 1.10. Experiment and Results

In order to verify the effectiveness of the method, the traditional IGA, the interactive genetic algorithm with graphical interaction mechanism (IGA-GIM), the interactive genetic algorithm with the K-D tree surrogate model (IGA-KDT), and the interactive genetic algorithm with the K-D tree surrogate model and graphical interaction mechanism (IGA-KDTGIM) are compared with each other. The evolution parameters of the four methods are all set as the same, the initial population size of the evolution parameters is set to 6, the crossover probability is 0.9, and the mutation probability is 0.1. Evolutionary operators include stochastic universal sampling and elite strategies, two-point crossover, and single-point mutation. The four methods have been independently operated by 10 users once, and the users have operated through the above interactive interface, and the population evolution was terminated after the 20th generation. This study mainly compares the experimental results in three aspects: the average fitness, average maximum fitness, and user evaluation times of the four algorithms, and the three aspects were compared through the same evolutionary generation, so as to compare the optimization capabilities of the algorithms and the ability of relieving user fatigue.

As experimental results, Figures 9 and 10 show a comparison of the fitness distributions of 10 users using the four methods.  Figure 9 shows a trend chart of the average fitness of each generation of evolutionary individuals. The four curves represent the trend of the average fitness of each generation of IGA, IGA-GIM, IGA-KDT, and IGA-KDTGIM in this paper. It can be seen from Figure 9 that the average fitness of the proposed algorithm increases with the increase of generation, and the fitness is much better than the comparison algorithm after the 10th generation. In the first 10 generations, there was no significant difference between IGA-KDT and IGA-KDTGIM in average fitness, and both of them were higher than IGA and IGA-GIM because the K-D tree surrogate model was used to assist users' evaluation and reduce users' evaluation noise, so as to improve fitness. In the last 10 generations, due to the use of GIM, the average fitness of IGA-KDTGIM and IGA-GIM has been significantly improved, but IGA-KDTGIM has a higher fitness due to the use of the surrogate model.  Figure 10 shows the trend of the average maximum fitness of evolutionary individuals. Obviously, the average maximum fitness of IGA-KDTGIM is higher than that of the other three methods. Therefore, K-D tree surrogate model and graphic interaction mechanism are effective in reducing users' evaluation noise, improving population quality, and accelerating users' search for satisfactory solutions.

Figure 11 shows the distribution of average fitness of four users who have used the proposed method. In the graph, the four curves show a general upward increasing trend, but there are still some minor local differences. Their fitness in the first generation is lower than 4 points, and it is higher than 6 points in the last generation. The reason is that this method combines user's evaluation of individual information and user's graphic interaction, which also proves the effectiveness of this method. User 1 curve is relatively flat and increasing, and user 2 curve is more variable and there are ups and downs in the mean fitness as a result of the randomness of gene locus crossover mutation. Therefore, the average fitness will have some peaks in the changing process, such as the 4th and 8th generations of user 2.

The results will be different according to the user's location of graphic interaction. Among the test users, user 1 and user 2 both have performed graphic interactive operations in the 11th generation, while user 3 and user 4 have performed graphical interactive operations in the 16th generation. It can be observed that the average fitness of all four users of the generated positions interacting with graphics has increased, but by contrast, the final average fitness of user 3 and user 4 is lower because the graphic interaction mechanism can bring the evolving population production more features that are satisfactory to users and can improve the average fitness of the population through multiple evolutions.

In this experiment, in order to verify that the K-D tree surrogate model reduces the evaluation times of users, the evaluation times of users have been recorded in the evolution process.  Figure 12 shows the evaluation times of users of the four algorithms. Obviously, the number of users' evaluations of IGA-KDT and IGA-KDTGIM is much lower than that of IGA and IGA-GIM, and the number of users' evaluations of the two algorithms is basically the same. This is because both methods use the K-D tree agent model to assist user evaluation, so as to reduce the number of user evaluation.

## 2. Conclusion

In this paper, the aim is to realize the intelligence and visualization of product design. This research proposes a method to improve IGA by using the K-D tree surrogate model and graphic interaction mechanism and thus builds a 3D vase modeling design system based on this method. This method uses the historical data of users to train the K-D tree surrogate model, searches for similar individuals through the nearest neighbor, provides a reference for users to evaluate individual fitness, and constantly updates the surrogate model to ensure the accuracy of prediction. In order to improve the efficiency of evolution, a graphic interaction mechanism has been introduced, through which users can dynamically change the individual shape, so as to help users increase the feature of individual satisfaction, expand the search space of the algorithm, and increase the diversity of the population. Experimental results show that this method has advantages in reducing the fatigue of users and speeding up the search for solutions to satisfy customers.

The application scope of the proposed algorithm is suitable for the target features to be well presented, and the specific feature boundary value and precision of the optimization target should be defined. Compared with the previous IGA methods, the proposed method is easier to obtain satisfactory solutions from users because it uses GIM in the interactive mode and shows better evolutionary optimization ability. In the future work, the IGA-KDTGIM will be used in the modeling design of other ceramic products.

## Figures and Tables

**Figure 1:** K-D tree data partition. (a) The first division of space. (b) The second division of space. (c) The third division of space. (d) The 20th division of space and search point.

**Figure 2:** Graphical interactive interface.

**Figure 3:** Flowchart of our algorithm.

**Figure 4:** Crossover and mutation.

**Figure 5:** Vase surface mesh model.

**Figure 6:** Vase model with texture mapping.

**Figure 7:** Cubic Bezier curve.

**Figure 8:** System interactive interface.

**Figure 9:** Comparison of the average fitness of evolved individuals.

**Figure 10:** Comparison of the average maximum fitness of evolved individuals.

**Figure 11:** Average fitness distribution of four users using the proposed method.

**Figure 12:** Comparison of user evaluation times of the four algorithms.

**Algorithm 1:** Details of algorithm steps.

## Data Availability

The data used to support the findings of this study are available from the corresponding author upon request.
